# ShenKang Injection Attenuates Renal Fibrosis by Inhibiting EMT and Regulating the Wnt/*β*-Catenin Pathway

**DOI:** 10.1155/2022/9705948

**Published:** 2022-06-28

**Authors:** Hui-Ting Wei, Yuan Xu, Xiao-Yang Tan, Hao-Yue Jing, Yue-Rong Ma

**Affiliations:** School of Basic Medicine, Chengdu University of Traditional Chinese Medicine, Chengdu 611137, China

## Abstract

Shenkang Injection (SKI) is a traditional Chinese medicine injection commonly used in the clinical treatment of chronic kidney disease. Although it has been confirmed that SKI has anti-kidney fibrosis effects, the underlying mechanism remains unclear. To investigate the effects of SKI on epithelial-mesenchymal transition (EMT) and Wnt/*β*-catenin pathway and explore its potential anti-fibrosis mechanism. A unilateral ureteral obstruction (UUO) model was induced by ligating the left ureter of male SD rats. A total of 24 rats were randomly divided into the following four groups: sham group, model group, SKI group, and benazepril group. The rats in each group were treated for 28 days, and renal function was evaluated by blood urea nitrogen (BUN) and serum creatinine (Scr). The degree of renal fibrosis was assessed by hematoxylin and eosin (HE) and Masson staining. Extracellular matrix (ECM) deposition was evaluated by immunohistochemistry. Real-time fluorescent quantitative PCR (RT-qPCR) and western blotting were used to detect the expression of genes and proteins in the Wnt/*β*-catenin signaling pathway. Further studies were performed in vitro using HK-2 cells treated with TGF-*β*1. At 28 days postoperation, the levels of BUN and Scr expression were significantly increased in the UUO group. SKI and benazepril reduced the levels of BUN and Scr, which displayed protective renal effects. Pathological staining showed that compared with the sham operation group, the renal parenchymal structure was severely damaged, the number of glomeruli was reduced, and a large amount of collagen was deposited in the kidney tissue of the UUO group. SKI treatment reduced morphological changes. Immunohistochemistry showed that compared with the sham operation group, the content of collagen I and FN in the kidney tissue of the UUO group were significantly increased, whereas the SKI content was decreased. In addition, compared with the UUO group, the levels of Wnt1, active *β*-catenin, Snail1, and PAI-1 expression were reduced in the SKI group, suggesting that SKI may reduce renal fibrosis by mediating the Wnt/*β*-catenin pathway. Further in vitro studies showed that collagen I, FN, and *α*-SMA levels in HK-2 cells were significantly increased following stimulation with TGF-*β*1. SKI could significantly reduce the expression of collagen I, FN, and *α*-SMA. A scratch test showed that SKI could reduce HK-2 migration. In addition, by stimulating TGF-*β*1, the levels of Wnt1, active *β*-catenin, snail1, and PAI-1 were significantly upregulated. SKI treatment could inhibit the activity of the Wnt/*β*-catenin signaling pathway in HK-2 cells. SKI improves kidney function by inhibiting renal fibrosis. The anti-fibrotic effects may be mediated by regulation of the Wnt/*β*-catenin pathway and EMT inhibition.

## 1. Introduction

Renal fibrosis is a common end-stage pathology associated with various chronic kidney diseases (CKD) and is expected to become the fifth leading cause of death in the world by 2040 [1]. Therefore, targeting renal fibrosis is considered to represent an important treatment strategy for CKD patients; however, there are currently no therapeutic drugs for renal fibrosis [2].

Renal fibrosis has complex etiology and pathogenesis, among which the epithelial-mesenchymal transition (EMT) of renal tubular epithelial cells is one of the most important mechanisms involved in renal fibrosis. Renal epithelial cells are transformed from mesenchymal-to-epithelial transition (MET) during embryonic development [3, 4]. It was not until a groundbreaking study in 2014 that it was recognized that epithelial cells could be converted into a mesenchymal phenotype through EMT, which impacted the understanding that epithelial cells always retain their properties until they die [5]. EMT was first described in embryogenesis [5] and subsequently observed in inflammation [6], fibrosis [7–9], wound healing [10], and cancer progression [11–13]. EMT in the kidney is an orchestrated process consisting of the classical four steps: loss of epithelial cell adhesion, destruction of the basement membrane, *α*-SMA synthesis, as well as cellular migration and invasion [14]. It is believed that epithelial cells injured via EMT could serve as an important source of fibroblasts, contributing to kidney fibrosis. Furthermore, EMT can significantly contribute to interstitial excessive extracellular matrix (ECM) deposition and promote the progression of renal fibrosis [15]. Therefore, improving EMT is considered to represent an important treatment strategy for patients with renal fibrosis.

The Wnt/*β*-catenin pathway is an indispensable, evolutionarily conserved pathway involved in the process of nephron formation. In normal adult kidneys, the Wnt/*β*-catenin pathway is quiescent and can be reactivated following kidney injury [16–19]. This continuous activation state is both harmful and also closely related to renal fibrosis. Several comprehensive reviews [20, 21] have emphasized the key role of this approach. *β*-catenin is a multifunctional cytoskeletal protein that exists in several different cell types, including endothelial cells, fibroblasts, and osteoblasts, in which it regulates their proliferation, differentiation, and apoptosis [22, 23]. Moreover, abnormal *β*-catenin expression is associated with CKD [16–18, 24, 25]. When kidney injury-induced *β*-catenin is activated, it serves as an effector molecule to amplify Wnt signaling. In *β*-catenin dephosphorylation, the free *β*-catenin was accumulated, and epithelial integrity was destroyed [26]. Therefore, focusing on a blockade of the Wnt/*β*-catenin signaling pathway may represent a potential treatment strategy for renal fibrosis.

Shenkang injection (SKI) is composed of four traditional Chinese herbs: *Astragalus mongholicus* Bunge, *Rheum officinale* Baill, *Salvia officinalis* L, and *Carthamus tinctorius* L. Moreover, SKI was developed from “Shenkang formula (SKF),” which was first used by Professor Chuan-hui Ye. SKI has been widely used clinically to treat chronic kidney disease [27]. Studies have shown that SKI can improve renal function in patients with renal failure. [28–30]. In addition, it has been demonstrated that SKI could block the pericyte-myofibroblast transition (PMT) by inhibiting platelet-derived growth factor receptor (PDGFR) activation and vascular endothelial growth factor receptor (VEGFR) signaling in the kidneys of unilateral ureteral obstruction (UUO) model rats [31]. SKI could provide protection against HG-induced renal tubular cell senescence for the treatment of diabetic nephropathy [32]. In addition, SKI could also reduce and alleviate diabetic tubulopathy (DT) in a similar manner as rosiglitazone and achieve this effect by inhibiting EMT and endoplasmic reticulum stress-induced apoptosis [33]. Moreover, SKI inhibits renal fibrosis and oxidative stress by downregulating the TGF-*β*/Smad3 signaling pathway in 5/6 nephrectomy [30]. However, the anti-fibrotic mechanism of SKI remains unknown. This study aimed to elucidate the anti-fibrotic effect of SKI by focusing on the Wnt/*β*-catenin signaling pathway. In particular, the effect of SKI on rat renal tissue fibrosis and HK-2 cellular trans-differentiation was observed, for which the clinical application of SKI in anti-kidney fibrosis treatment provides evidence.

## 2. Materials and Methods

### 2.1. Animals

A total of 50 eight-week-old male SD rats weighing 210 g ± 20 g, were purchased from Chengdu Dashuo Experimental Animal Co. Ltd. The rats were raised in separate cages at the Animal Experiment Center of Chengdu University of Traditional Chinese Medicine. The temperature was controlled at 20°C–25°C; the humidity was maintained at 50%–60%; and a density of six rats per cage. Rats were free to eat and drink for a week. The study was conducted under the guidance of the Ethics Committee of Chengdu University of Traditional Chinese Medicine. Every effort was made to reduce animal suffering.

### 2.2. Animal Model Inducing Renal Fibrosis

Rats underwent a unilateral ureteral obstruction (UUO) operation. The experiment was completed under aseptic conditions, and the specific UUO steps were performed as follows: the rats were placed in the supine position after anesthesia. A longitudinal incision was made 1 cm next to the midline of the abdomen. The left kidney was located; the surrounding fat tissue was peeled off; the ureter was freed; and the upper 2/3 section of the ureter was ligated with a 4-0 surgical silk suture and ligated again approximately 5 mm apart to ensure the success of the model [34, 35]. A total of 33 surviving rats were randomly divided into three groups: the model group, SKI group, and Benazepril group (*n* = 11 per group). In the sham group, only the left kidney was exposed during the operation. The dose of SKI was administered to rats at a dose of 0.9 mL/day, which was half the equivalent dose for clinical use. Benazepril rats were administered at a clinically therapeutic equivalent dose of 0.9 mg/kg. Benazepril was dissolved in distilled water into a 1 mL suspension for intragastric administration. After treatment for 28 days, 24 rats in the sham group, model group, SKI group, and benazepril group (6 per group) survived and were included in the group for data analysis.

### 2.3. Drug Preparation

SKI was purchased from Xi'an Century Shengkang Pharmaceutical Co. Ltd. The batch number was 202012113 and contained the following four traditional Chinese medicine extracts: Safflower, Rhubarb, *Astragalus*, and Salvia. The medical extraction and preparation of SKI obtained Chinese patent certification and protection. In the same batch, the main components were subjected to standardization. Each 20 mL SKI contained 6 g of raw medicine, and the equivalent dosage of SKI was 1.8 mL/day. Each dosage of SKI was prepared in a 0.9 mL/d liquid for the administration of an intraperitoneal injection. In preliminary experiments, three drug concentrations were selected: high (3.6 mL/d), medium (1.8 mL/d), and low (0.9 mL/d). The effect of the high-dose treatment effect was not good, and both the middle- and low-dose treatment effect was equivalent. Finally, the low dose was selected for further research into its therapeutic effect. Both fingerprint and chromatographic analyses were conducted to perform a chemical and quantitative analysis of SKI [36, 37]. Benazepril hydrochloride tablets were produced by Chengdu Diao Pharmaceutical Group Co. Ltd. and purchased from the Affiliated Hospital of the Chengdu University of TCM.

### 2.4. Scr and BUN Assessment of Renal Function

A veterinary biochemical analyzer was used to detect serum creatinine, 28 days after the operation (Shenzhen Mindray Biomedical Electronics Co. Ltd., BS-240VET). BUN was tested using a commercial kit (Nanjing Jiancheng Institute of Biological Engineering, C013-2-1). The rat body weight and kidney weight were also measured with an electronic scale (i2000) and electronic balance (HANGPING JA3003) 28 days postoperatively, respectively.

### 2.5. Histopathological Examination of the Kidney

The kidney was cut vertically into two parts along the largest longitudinal section. One half was fixed with 10% formaldehyde, and the renal tissue was processed by hematoxylin-eosin (HE) and Masson staining. The pathological sections were observed under a microscope (ECLIPSE Ni-E Nikon, Tokyo, Japan). HE staining was used to count the number of glomeruli. A total of 10 separate views (100×) of the HE stained sections were selected, and the number of glomeruli was counted. A total of 6 separate views (100×) of the Masson stained sections were selected to evaluate the degree of renal fibrosis. The collagen volume fraction (CVF) was analyzed using ImageJ software.

### 2.6. Cell Culture

The normal human kidney immortalized proximal tubule epithelial cell line, HK-2 cells, were purchased from the Shanghai Cell Bank of the Chinese Academy of Sciences (Shanghai, China) and cultured in DMEM supplemented with 10% fetal bovine serum (FBS) and 1% penicillin-streptomycin solution at 37°C in a 5% CO_2_ incubator. Under the microscope, the cells were adherent. TGF-*β*1 is a known fibrosis inducer, and ICG-001 is a known Wnt/*β*-catenin pathway inhibitor; thus, TGF-*β*1 could be used to induce EMT in HK-2 cells. ICG-001 can be used in rescue experiments to further confirm the role of the Wnt/*β*-catenin pathway in renal fibrosis. TGF-*β*1 was obtained from Abcam (ab50036), and ICG-001 was purchased from AbMole (M2008). To investigate the role of SKI in cell EMT, HK-2 cells were treated with TGF-*β*1 (10 ng/mL) for 24 h at 37°C. HK-2 cells in the exponential growth phase were digested with 0.25% trypsin-EDTA, passaged, and counted, and the HK-2 cells were inoculated into a six-well plate. Next, either SKI or ICG-001 was mixed with TGF-*β*1. After 24 h of stimulation, the cells were collected for further analysis.

### 2.7. CCK-8 Assay

CCK-8 was used to select the appropriate concentration of SKI drugs. HK-2 cells were seeded into each well of a 96-well plate at a density of 6 × 10^3^ cells/well. After overnight incubation at 37 C, the samples were divided into a control group and an experimental group. The control group was cultured normally, whereas the experimental group was treated with 10, 5, 2.5, 1.25, and 0.75 mL SKI. Next, CCK-8 reagent and serum-free solution (1 : 10) medium were added to each well, followed by incubation for 1 h at 37°C in 5% CO_2_. A VARIOSKAN microplate reader (Thermo Electronics Corporation) was used to quantify the optical density (OD) at 450 nm.

### 2.8. Scratch Test

Cell motility was assessed by a wound healing measurement. The cells were cultured in six-well plates (10 × 10^4^ cells/well). At 80%–90% confluency, the cellular monolayer was scraped with a sterile 200 *μ*L suction head and cultured under standard conditions for 24 h. Wound healing was captured at 0 h and 24 h under a microscope, and the scratch ratio was calculated using the following formula: acratch ratio = (area 0 h – area 24 h)/area 0 h.

### 2.9. Phalloidin Staining

For fluorescence staining with phalloidin, HK-2 cells were plated into a 12‐well plate. Staining was performed using Actin-Tracker Green (FITC) labeled phalloidin (Beyotime Biotechnology Co. Ltd., Shanghai, China; lot number: C1033) in accordance with the manufacturer's instructions. The labeled cells were analyzed using a Nikon ECLIPSE Ti (606208, Japan).

### 2.10. Immunohistochemical (IHC) Examination

Collagen I, FN, *α*-SMA, and E-cadherin were detected using IHC. The steps are as follows: paraffin sectioning, deparaffinization, antigen recovery, and serum blocking. The primary antibody of the target protein (Table 1) was added and incubated overnight at 4°C. The corresponding secondary antibodies (HRP rabbit anti-goat IgG (*H* + *L*; AS029, 1 : 500) and HRP donkey anti-mouse IgG (*H* + *L*; AS033, 1 : 500) were added after washing. SABC was added and washed again, and DAB was added for color development and dehydration and mounted after counterstaining. Six individual sections were randomly selected to calculate the integrated optical density.

### 2.11. Immunofluorescence (IF) Examination

The cultured HK-2 cells were fixed with 4% paraformaldehyde and washed three times with 0.1% Triton X-100. The cells were combined with preconfigured anti-E-cadherin (Abcam ab231303, 1:1,000), anti-*α*-SMA (Abclonal A17910, 1:200), and active *β*-catenin (CST 8814, 1:1,000) antibodies and incubated with primary antibodies at 4°C overnight. The cells were incubated with the corresponding secondary antibody for 1 h at room temperature. Mouse (FITC goat anti-mouse IgG (*H* + *L*); AS001, 1:50) or rabbit (FITC goat anti-rabbit IgG (*H* + *L*); AS011, 1:50) antibodies were incubated with secondary antibodies. DAPI was used to counterstain the cell nucleus, and an anti-fluorescence quencher was added and was mounted on a glass slide. HK-2 cells were observed under Nikon ECLIPSE Ti (606208, Japan).

### 2.12. Real-Time Fluorescence Quantitative PCR (RT-qPCR)

The total RNA was extracted using an animal total RNA isolation kit (RE-03011 FOREGENE, Biologix, Camarillo, CA, USA). A ScanDrop 100 was used to detect the level of RNA purity. cDNA was synthesized using a Master PremixRT EasyTM II (RE-01022 FORE GENE). qPCR (qTower3G, Germany) displayed the following thermal cycle curve: 95°C for 3 min, 95°C for 10 s, and 40 amplification cycles (95°C for 10 s, 65°C for 30 s, and 60°C for 15 s). The reaction system consisted of 20 *μ*L, including 6.4 *μ*L DNase-free (dd) water, 10 *μ*L Mix SYBR (QP-01014 FOREGENE), 0.8 *μ*L forward and reverse primers, and 2 *μ*L cDNA diluent. The absorbance of SYBR green fluorescence was detected in each tube at the end of each cycle. The cycle threshold (CT) values were obtained. The primers used in this study are shown in Table 2. The target genes included collagen I, FN, *α*-SMA, E-cadherin, Wnt1, PAI-1, *β*-catenin, and Snail1. The primers were supplied by Tsingke Biotechnology Co. Ltd. The relative expression values of the target genes were calculated using the 2^−ΔΔCt^ method [38].

### 2.13. Western Blot

The renal tissue was homogenized in radioimmunoprecipitation assay (RIPA) protein lysate containing protease and phosphatase inhibitors. After centrifugation (12,000 rmp, 5 min), the supernatant was retained, and its total protein content was determined according to the bicinchoninic acid (Beyotime Biotechnology Co. Ltd., Shanghai, China; lot number: P0012) kit instructions. A 5 × SDS-PAGE loading buffer was used to balance the loading volume of each well to 40 mg/10 mL. Next, 5 × protein loading buffer was added to each sample solution, mixed well, boiled at 100°C for 15 min, cooled, and stored at −20°C until subsequent use. The samples were subjected to 10% SDS-PAGE gel, and the separated proteins were transferred to polyvinylidene fluoride (PVDF) membranes (1212639 GVS, Sanford, ME, USA). The membranes were blocked in phosphate-buffered saline Tween 20 (PBST) containing 5% bovine serum albumin (BSA) at room temperature for 1.5 h. Primary antibodies were incubated with the membranes at 4°C for 12 h, after which the membrane was incubated with the secondary antibody at room temperature for 1.5 h. The immunoreactive protein bands were visualized using ECL (NcmECL Ultra, NCM Biotech) chemiluminescence method for color rendering. An E-blot electronic tablet imager was used for membrane visualization and analysis (Shanghai E-Bote Optoelectronics Technology Co. Ltd., Shanghai, China). The final reported data for collagen I, *α*-SMA, E-cadherin, Wnt1, PAI-1, *β*-catenin, active-*β*-catenin, and Snail1 were the results of the relative internal reference proteins. The primary antibodies used in this study are shown in Table 1.

### 2.14. Statistical Analysis

Continuous data were expressed as the mean ± standard deviation. A one-way analysis of variance (ANOVA) was used for comparisons among multiple groups, and the least significant difference-t test (LSD-t test) was used for pairwise comparisons. A threshold of *P* < 0.05 indicated a statistically significant difference. SPSS 20.0 statistical software (IBM Corp., Armonk, NY, USA) was used for data analysis.

## 3. Results

### 3.1. SKI Improves the Renal Function of UUO Rats

The renal function of rats reacted by BUN and Scr (Figures 1(a) and 1(b)). The levels of BUN and Scr in the UUO group were significantly higher compared with those in the sham group (*P* < 0.001). The wet weight of the left kidney was significantly increased (Figure 1(c); *P* < 0.001). After SKI treatment, the levels of BUN and Scr in the rats were significantly lower than those in the UUO group (*P* < 0.001), and the wet weight of the left kidney was mildly decreased (*P* < 0.05). These results indicate that SKI can improve the renal function impaired by UUO surgery.

### 3.2. SKI Attenuates ECM Deposition in UUO Rats

Rat HE-stained renal tissue exhibited a normal, organized architecture in the sham group; however, in the UUO group, the number of glomeruli was decreased, renal tubular displayed atrophy, some tubules and collecting ducts were dilated, and tubular epithelial cells were vacuolated; interstitial fibroblasts were proliferated, and extensive inflammatory cells were infiltrated (Figure 2(a)). The number of glomeruli was counted by randomly selecting 10 views for each section HE stained under 100 × magnification (Figures 2(b) and 2(c)). Compared with the sham group, the number of glomeruli in the UUO group decreased to 36.33 (*P* < 0.001). In addition, the number of glomeruli was increased to 51.33 (*P* < 0.05) following SKI treatment. Benazepril exhibited similar effects to that of SKI. Masson staining revealed extensive collagen deposition in the UUO group; however, SKI treatment greatly reduced the amount of collagen deposition in UUO rats (Figure 2(d)). The collagen volume fraction (CVF) was used to indirectly reflect changes in collagen deposition (Figure 2(e)). The CVF of the model group was 4.67 times higher than that of the sham operation group (*P* < 0.001). After SKI treatment, CVF was decreased by 58.14% (*P* < 0.001). The level of collagen I and FN expression in the kidney tissue was evaluated by immunohistochemical methods (Figures 3(a) and 3(b)). Compared with the sham group, the integrated optical density (IOD) of collagen I and FN (Figures 3(c) and 3(d)) in the UUO group increased to 14% and 24%, respectively (*P* < 0.001). After SKI treatment, the IOD of type I collagen and FN decreased to 12% and 19% (*P* < 0.001). Compared with the UUO group, the level of collagen I protein expression, *Col1a1*, and *Fn1* mRNA expression in the SKI group was also decreased (Figures 3(e)–3(h)). These results indicate that SKI could effectively reduce renal fibrosis by inhibiting the expression and deposition of ECM. Similar effects were observed in the Benazepril group.

### 3.3. Effects of SKI on EMT in UUO Rats

EMT, including the loss of cell-cell adhesion, apical-basal polarity, and mesenchymal characteristics, which confer migratory capacity were acquired. The downregulation of E-cadherin expression and upregulation of some mesenchymal genes are characteristics of EMT. Immunohistochemistry was used to assess the contents of *α*-SMA and E-cadherin in the renal tissue (Figures 4(a) and 4(b)). The IOD of *α*-SMA (Figure 4(c)) was significantly reduced in the SKI group (*P* < 0.001), whereas the IOD of E-cadherin (Figure 4(d)) was increased (*P* < 0.001). Compared with the UUO group, the level of *Acta2* RNA and protein expression in the SKI group were also reduced (Figure 4(e), 4(f), and 4(h)). The opposite effect was observed in the level of E-cadherin (*Cdh1*) RNA and protein expression (Figures 4(e), 4(g), and 4(i)). Benazepril showed similar effects to that of SKI. These results indicate that SKI could effectively reduce renal fibrosis by restraining EMT.

### 3.4. SKI Downregulated the Wnt/*β*-Catenin Signaling Pathway in the Renal Tissue of UUO Rats

The Wnt/*β*-catenin signaling pathway is considered to be closely related to renal fibrosis. The effects of SKI on the Wnt/*β*-catenin signaling pathway in the renal tissue of UUO rats were investigated. Compared with the sham operation group, Wnt1 (*P* < 0.01), *β*-catenin (*P* < 0.001), active *β*-catenin (*P* < 0.01), Snail1 (*P* < 0.001), PAI-1 (*P* < 0.01), and TCF4 (*P* < 0.001) protein expression were significantly increased (Figures 5(a)–5(g)). The expression of Wnt1, *β*-catenin, active *β*-catenin, Snail1, PAI-1, and TCF4 was measured by RT-qPCR and/or western blot. The results showed that the mRNA expression of *Wnt1*, *Ctnnb1*, *Serpine1*, *Snail1*, and *Tcf4* in the UUO group (Figures 5(h)–5(l)) was significantly increased (*P* < 0.001). SKI treatment could reduce the level of Wnt1 (*P* < 0.01), *β*-catenin (*P* < 0.001), active *β*-catenin (*P* < 0.05), Snail1 (*P* < 0.01), PAI-1 (*P* < 0.05), and TCF4 (*P* < 0.01) expression.

### 3.5. The Effect of SKI on HK-2 Cells Stimulated with TGF-*β*1

The effect of SKI on HK-2 cells stimulated by TGF-*β*1 was further studied. The model group of HK-2 cells was cultured in DMEM with 10 ng/mL TGF-*β*1, and the treatment group was administered SKI on this basis. RT-qPCR and/or western blot were used to detect the levels of collagen I and FN. The results showed that compared with the cells cultured in DMEM, the cells secreted more *Col1a1* and *Fn1* following treatment with TGF-*β*1 (*P* < 0.001 and *P* < 0.001, respectively; Figures 6(a), 6(b), 6(e), and 6(f)). SKI treatment significantly reduced the levels of collagen I and FN (Figures 6(a), 6(b), 6(e) and 6(f)). Collectively, SKI could effectively inhibit collagen I and FN production in HK-2 cells. TGF-*β*1 is the most potent factor triggering EMT in renal cells. According to a popular perspective, EMT represents a process by which epithelial cells escape from the unfavorable microenvironment under conditions of stress. *α*-SMA is characteristically expressed in interstitial cells around injured tubules and myofibroblasts. The decrease or loss of epithelial cell markers (e.g., E-cadherin) is strongly suggestive of EMT. The results showed that (Figures 6(a), 6(c), and 6(g)) *α*-SMA expression was upregulated and E-cadherin (Figures 7(a), 7(d), and 7(h)) expression was decreased in TGF-*β*1-stimulated cells. SKI inhibited the expression of *α*-SMA and promoted the expression of E-cadherin. The scratch test validated that cells treated with TGF-*β*1 exhibited significant migration, whereas SKI improved HK-2 cell migration owing to the treatment of TGF-*β*1 (Figures 8(a) and 8(b)). The scratch ratio in the cells treated with TGF-*β*1 was increased to 0.85 (*P* < 0.001), compared with cells treated with DMEM. The scratch ratio was downregulated to 0.33 (*P* < 0.001) in the treatment with SKI (Figure 8(c)). Phalloidin staining was performed to intuitively reflect the phenotypic changes brought about by EMT. Phalloidin staining showed that cells treated with DMEM displayed a normal organized architecture, while spindle-shaped changes could be observed in cells stimulated by TGF-*β*1 (Figure 8(d)). SKI significantly inhibited these changes. These data suggest that SKI could restrain EMT in TGF-*β*1-stimulated HK-2 cells.

### 3.6. SKI Regulated TGF-*β*1-Activation of the Wnt/*β*-Catenin Signaling Pathway in HK-2 Cells

In vitro studies further confirmed the influence of SKI on the Wnt/*β*-catenin signaling pathway. TGF-*β*1-stimulated HK-2 cells were treated with SKI and the Wnt/*β*-catenin signaling pathway inhibitor, ICG-001, for 24 h. The levels of collagen I, FN, *α*-SMA, and E-cadherin were measured in the same manner as described previously. Scratch test was also performed as described above. ICG-001 showed similar effects to that of SKI.

After inhibiting the Wnt/*β*-catenin pathway, immunofluorescence staining demonstrated that the level of *α*-SMA protein expression was inhibited, while E-Ca protein expression was upregulated by SKI (Figure 7(a)). RT-qPCR and/or western blot results showed that *α*-SMA (Figures 7(b), 7(d), and 7(f)) expression was decreased and E-cadherin (Figures 7(b), 7(e), and 7(g)) expression was upregulated in ICG-001 treated cells. The expression levels of collagen I and FN decreased (Figures 7(b), 7(c), 7(h), and 7(i)). The scratch ratio was also downregulated (*P* < 0.001) in the treated with ICG-001 (Figures 9(a)–9(c)). As shown by immunofluorescence, the cells treated with TGF-*β*1 showed significantly higher *β*-catenin expression (Figure 10(a)). The expression of Wnt1 (*P* < 0.01), *β*-catenin (*P* < 0.01), active *β*-catenin (*P* < 0.001), Snail1 (*P* < 0.001), PAI-1 (*P* < 0.01), and TCF4 (*P* < 0.01) were dramatically increased compared with the cells cultured with DMEM (Figure 10(b)–10(h)). SKI could reduce the level of Wnt1 (*P* < 0.05), *β*-catenin (*P* < 0.01), active *β*-catenin (*P* < 0.05), Snail1, PAI-1 (*P* < 0.05), and TCF4 (*P* < 0.05) mRNA (Figure 10(i)–10(m)). The level of mRNA expression showed similar results. The Wnt/*β*-catenin signaling pathway inhibitor, ICG-001, suppressed the expression of *β*-catenin, active *β*-catenin, Snail1, PAI-1, and TCF4, whereas it had no influence on Wnt1 (*P* > 0.05). These results confirmed that SKI could reduce fibrosis by inhibiting the Wnt/*β*-catenin signaling pathway.

## 4. Discussion

Renal fibrosis represented the major hallmark of nearly all progressive chronic kidney diseases. EMT was first discovered to be associated with fibrogenesis in renal tubular epithelial cells of a mouse anti-tubular membrane disease model [39]. The mouse renal fibrosis model induced by unilateral ureteral obstruction also confirmed that fibroblasts may be derived from transformed epithelial cells [22]. The concept and mechanism of EMT remain controversial. The definition of EMT did not consider the transformation of epithelial cells into any specific cell type but was defined by the phenotypic and functional changes associated with reminiscent mesenchymal cells. In renal fibrosis, epithelial cells migrate from the tubular structure into the interstitium and produce a matrix, thereby acting as new fibroblasts. Therefore, improving EMT and reducing ECM deposition represent a potential treatment for chronic kidney disease. SKI has been clinically used to delay the progression of renal failure, and animal studies have shown that SKI has anti-fibrotic effects [29, 30]. Our research confirmed that UUO surgery can induce renal fibrosis and impair renal function. Histopathology showed that a large amount of ECM was extensively deposited in the renal interstitium, and there was a significant reduction in the number of glomeruli. After 28 days of SKI treatment, the ECM deposition was significantly decreased; the number of glomeruli increased; and renal function recovered, all of which suggested that SKI can reduce renal fibrosis. In vitro studies further explored the potential anti-fibrotic mechanism of SKI. In addition, SKI could inhibit the expression of collagen I, FN, and *α*-SMA in HK-2 cells, as well as reduce the migration of HK-2 cells treated with TGF-*β*1 and restore phenotypic changes. Thus, SKI may be related to EMT suppression.

The Wnt/*β*-catenin pathway is a canonical pathway involved in the progression of fibrosis. In addition, *β*-catenin is a multifunctional cytoskeletal protein, which forms a cell adhesion link complex with E-cadherin to achieve epithelial integrity. Wnt binds with the receptor in the plasma membrane to induce a destruction complex composed of GSK-3*β*, CK1, APC, Axin, and *β*-catenin changes. In addition, the phosphorylation of GSK-3*β* can activate *β*-catenin to mediate Wnt canonical signaling. The level of active *β*-catenin in the cytoplasm was increased and subsequently translocated into the nucleus where it combined with TCF/LEF to induce the transcription of fibrosis-related genes, including Snail1, PAI-1, and FN. Snail1 is a key transcription factor driving EMT, and it cannot only inhibit the expression of E-cadherin but also causes the destruction of epithelial cell-cell adhesion [9]. Studies have shown that Snail1 and *β*-catenin are upregulated in the renal tubular epithelium of human and animal fibrotic kidneys [16, 40]. In vitro studies revealed that *β*-catenin activation induces Snail1 expression in both renal tubular epithelium cells and podocytes. PAI-1 participates in inflammation and plays a vital role in the pathogenesis of fibrogenesis, and FN is a component of ECM. In addition, other genes (e.g., *MMP-7* and *RAS*) also play a vital role in fibrogenesis. SKI can improve renal function and inhibit *β*-catenin, Snail1, PAI-1, TCF4, and Wnt1 expression. Our results show Wnt/*β*-catenin signaling pathway activation in HK-2 cells following stimulation with TGF-*β*1, which resulted in the production of active *β*-catenin. Active *β*-catenin promotes Snail1, PAI-1, and TCF4 expression. In addition, SKI can inhibit TGF-*β*1-induced activation of the Wnt/*β*-catenin signaling pathway in HK-2 cells and reduce *β*-catenin activity. Therefore, we speculate that SKI may play a role in inhibiting the activation of *β*-catenin.

## 5. Conclusion

In summary, our in vivo and in vitro research showed that SKI could improve renal function and exhibit anti-fibrotic effects. The underlying mechanism might be related to inhibiting the Wnt/*β*-catenin signaling pathway. *β*-catenin may represent an attractive treatment target for renal fibrosis, and improving EMT may have favorable anti-fibrosis effects. This research provides basic mechanistic support for the clinical application of SKI.

## Figures and Tables

**Figure 1:** Treatment with SKI improved kidney function: (a) the level of BUN expression, (b) the level of Scr was determined using an automatic biochemical analyzer, and (c) the rat kidney wet weight.

**Figure 2:** Treatment with SKI attenuated the renal lesions and fibrosis caused by UUO: (a) kidney sections of the four groups were subjected to HE staining (400×), (b) HE staining (100 × for the glomeruli count), (c) the degree of renal fibrosis in renal tissue was analyzed to quantitatively assess the number of glomeruli, and (d and e) Masson staining (200×). The CVF was analyzed to quantitatively assess the collagen content in the renal tissue.

**Figure 3:** SKI reduces the ECM deposition caused by UUO: (a and c) immunohistochemical and IOD statistical analysis of FN, (b and d) immunohistochemical and IOD statistical analysis of Col1, (e) western blotting images of Col1 and actin, (f) relative level of Col1 protein expression in UUO rats, and (g and h) qRT-PCR revealed Col1 and FN mRNA expression.

**Figure 4:** SKI improves EMT in the renal fibrosis of UUO rats: (a and c) immunohistochemical and IOD statistical analysis of *α*-SMA; (b and d) immunohistochemical and IOD statistical analysis of E-Ca; (e) western blotting images of *α*-SMA, E-Ca, and actin; (f and g) relative level of *α*-SMA and E-Ca protein expression in UUO rats; and (h and i) qRT-PCR revealed the level of *α*-SMA and E-Ca mRNA expression.

**Figure 5:** SKI inhibited activation of the Wnt/*β*-catenin signaling pathway: (a) representative western blotting analyses, illustrating that SKI reduced the levels of, Snail1, TCF4, active *β*-catenin, *β*-catenin, PAI-1, and WNT1 protein expression, which are involved in the Wnt/*β*-catenin signaling pathway; (b–g) graphic presentation of Snail1, TCF4, active *β*-catenin, *β*-catenin, PAI-1, and WNT1 in the four groups as indicated; and (h–l) qRT-PCR revealed that SKI reversed the increased level of Snail1, Tcf4, Ctnnb1, PAI-1, and Wnt1mRNA expression.

**Figure 6:** SKI suppressed TGF-*β*1-induced HK-2 cell expression of *α*-SMA and production of collagen I and FN while upregulating E-cadherin expression: (a) western blotting images of *α*-SMA, E-Ca, Col1, and GAPDH; (b) the relative level of Col1 protein expression in HK-2 cells; (c and d) relative level of *α*-SMA and E-Ca protein expression in HK-2 cells; (e and f) qRT-PCR revealed the level of Col1 and FN mRNA expression; and (g and h) qRT-PCR revealed the level of *α*-SMA and E-Ca mRNA expression.

**Figure 7:** SKI-mediated EMT through inhibiting the Wnt/*β*-catenin signaling pathway: (a) immunofluorescence staining demonstrated that the level of *α*-SMA protein expression was inhibited while E-Ca protein expression was upregulated by SKI (200×); (b) western blotting images of Col1, *α*-SMA, E-Ca, and Actin; (c–e) the relative level of Col1, *α*-SMA, and E-Ca protein expression in HK-2 cells; and (f–i) qRT-PCR revealed the level of Col1, FN, *α*-SMA, and E-Ca mRNA expression.

**Figure 8:** SKI improved HK-2 cell migration in response to TGF-*β*1 treatment: (a) cell wound healing measurement at 0 h, (b) cell wound healing measurement at 24 h, (c) statistical analysis of the scratch test, and (d) fluorescence staining with phalloidin (400×). Phalloidin staining showed that cells treated with DMEM displayed a normal organized architecture, while spindle-shaped changes could be observed in cells stimulated by TGF-*β*1. Morphological changes alleviated after using SKI.

**Figure 9:** ICG-001 improved HK-2 cell migration in response to TGF-*β*1 treatment: (a) cell wound healing measurement at 0 h, (b) cell wound healing measurement at 24 h, and (c) statistical analysis of the scratch test.

**Figure 10:** SKI regulated TGF-*β*1-mediated activation of the Wnt/*β*-catenin signaling pathway in HK-2 cells: (a) immunofluorescence staining demonstrating that *β*-catenin protein expression was inhibited by SKI (200×); (b) western blotting images of active *β*-catenin, Snail1, TCF4, WNT1, *β*-catenin, and PAI-1, which are involved in the Wnt/*β*-catenin signaling pathway; (c–h) graphic presentation of active *β*-catenin, Snail1, TCF4, WNT1, *β*-catenin, and PAI-1 expression in the four groups as indicated; and (i–m) qRT-PCR revealed that SKI reversed the increased level of Snail1, Tcf4, Ctnnb1 (*β*-catenin), and PAI-1 mRNA expression.

**Table 1:** Primary antibody used in IHC and western blot experiment.

Protein	Primary antibody	Concentration
Collagen I	Abclonal; A16891	1 : 500
FN	Abcam; ab268021	1 : 2000
*α*-SMA	Abclonal; A17910	1 : 500
E-cadherin	Abcam; ab231303	1 : 1000
Collagen I	Abcam, ab260043	1 : 1000
Wnt1	Abclonal; A2475,	1 : 1000
*β*-catenin	Abclonal; A11512	1 : 1000
*β*-catenin (active)	Abcam; ab246540,	1 : 1000
PAI-1	Abcam; ab182973	1 : 1000
Snail1	Abclonal; A11794	1 : 500
Actin	Abclonal; AC026	1 : 200000
Gapdh	Abclonal; AC002	1 : 20000

**Table 2:** Primer sequences used in the qRT-PCR experiment.

Genes	Forward primers (5'⟶3')	Reverse primers (3'⟶5')
*Gapdh*	GGGCTGCCTTCTCTTGTGAC	CCCGTTGATGACCAGCTTCC
*Actb*	AGATCAAGATCATTGCTCCTCCT	ACGCAGCTCAGTAACAGTCC
*Wnt1*	CACCCTCATCCCAACTCACT	GGGGCGAAGAGCCACTAATA
*Tcf4*	CAGCCATTCTCTCCTGCCAA	GTAGGTTCTCATCGCCCTCG
*Fn1*	CTTACAACGTCAACGACACG	TGGGGTCACATTTCCATCTG
*Col1a1*	TCACTGCAAGAACAGCGTAG	AAGCGTGCTGTAGGTGAATC
*Ctnnb1*	ACCATCGAGAGGGCTTGTTG	CGCACTGCCATTTTAGCTCC
*Cdh1*	CTGGGGTCATCAGTGTGGTC	CTTGACCCTGGTACGTGCTT
*Acta2*	GGATCAGCGCCTTCAGTTCT	AGGGCTAGAAGGGTAGCACA
*Snai1*	GCTGCTTCGAGCCATAGAAC	TGTGTCCAGTTACCACCCTG
*Serpine1*	TCTTTCCGACCAAGAGCAGC	TGCGGGCTGAGACTAGAATG
*h-Gapdh*	GGAGTCCACTGGCGTCTTCA	GTCATGAGTCCTTCCACGATACC
*h-Actb*	TCCAAATATGAGATGCGTTGTTAC	TCCTTAGAGAGAAGTGGGGTG
*h-Wnt1*	CTTCGGCAAGATCGTCAACC	GCCGAAGTCAATGTTGTCGC
*h-Tcf4*	GATGCTCTGGGGAAAGCACT	AGCCAACAGGAGTTGAAGGG
*h-Fn1*	GGGAACACTTACCGAGTGGG	GCTTGCAGGTCCAATTCTCCT
*h-Col1a1*	GCTACTACCGGGCTGATGAT	TTGGTTGGGGTCAATCCAGT
*h-Ctnnb1*	CATGCACCTTTGCGTGAGCA	CCCCCTCCACAAATTGCTGC
*h-Cdh1*	AGGGGTTAAGCACAACAGCA	GGTATTGGGGGCATCAGCAT
*h-Acta2*	CTGAGCGTGGCTATTCCTTC	GTTTCATGGATGCCAGCAGA
*h-Snai1*	TAGCGAGTGGTTCTTCTGCG	AGGGCTGCTGGAAGGTAAAC
*h-Serpine1*	GGCTCAGACCAACAAGTTCA	GCAGTTCCAGGATGTCGTAG

## Data Availability

The data used to support the findings of this study are available from the corresponding author upon request.
